# The Application Value of SMI Technology and Contrast-Enhanced Ultrasound in the Differential Diagnosis of Benign and Malignant Thyroid Nodules

**DOI:** 10.1155/2022/6157026

**Published:** 2022-08-25

**Authors:** Jiahuan Wu, Tian Zhan, Honggang Sun, Fanbo Wang

**Affiliations:** ^1^Department of Neurology, The First Affiliated Hospital of Jiamusi University, Jiamusi 154000, Heilongjiang, China; ^2^Department of Neurology, 970 Hospital of Yantai Joint Logistics Support Force, Yantai 264000, Shandong, China; ^3^Department of Pathology, The First Affiliated Hospital of Jiamusi University, Jiamusi 154000, Heilongjiang, China; ^4^Physical Diagnosis Department, The First Affiliated Hospital of Jiamusi University, Jiamusi 154000, Heilongjiang, China

## Abstract

Thyroid disease has always been a common and frequent disease in clinical medicine, and its disease detection rate has been increasing year by year. Thyroid diseases are mainly divided into two categories: thyroid diseases treated by medical treatment and thyroid diseases treated by surgery. Thyroid cancer has also become one of the most common malignant secretory tumor diseases today. Ultrasound examination is a commonly used method for diagnosing thyroid diseases. During the diagnosis process, doctors need to observe the characteristics of ultrasound images and combine professional knowledge and clinical experience to give the patient's disease status. With the improvement of people's living standards and health awareness, thyroid disease has become an important issue that plagues the health of Chinese residents. Therefore, people and medical workers are paying more attention to thyroid disease. In recent years, various ultrasound technologies have been applied in the differential diagnosis of benign and malignant thyroid nodules and have played an important role in the diagnosis. This article aims to study the application value of SMI technology (ultra-microvascular imaging technology) and contrast-enhanced ultrasound in the differential diagnosis of thyroid benign and malignant nodules. It conducts diagnostic experiments and analysis on some cases of benign and malignant thyroid nodules through the use of SMI diagnostic methods and contrast-enhanced ultrasound examination methods. And the ROC curve was used to calculate the sensitivity of SMI technology and ultrasound for the identification and diagnosis of thyroid benign and malignant nodules, and the results were 0.83 and 0.81, respectively. It is concluded that SMI technology and contrast-enhanced ultrasound examination have good diagnostic efficiency and application value for the identification and diagnosis of thyroid benign and malignant nodules.

## 1. Introduction

The thyroid is an important organ of the human body, and it plays an important role in maintaining the health of the human endocrine system and the physical and mental health of the human body. With the advancement of medical ultrasound technology, ultrasound examination has become one of the most commonly used early detection methods for diseases due to its advantages such as low price, safety, noninvasiveness, convenient use, and ability to reflect the actual situation of tissues. A thyroid nodule refers to a mass in normal thyroid tissue that is different from normal glandular tissue. Thyroid nodules can be divided into two categories according to their nature: benign nodules and malignant nodules. Among them, benign nodules can be divided into nodular goiter, thyroid adenoma, and Hashimoto's thyroiditis; the main type of malignant nodules is thyroid papilloma, which is the most common pathological type with the highest incidence of malignant thyroid nodules, while other pathological types are relatively rare. Due to the superficial location of the thyroid, the boundary between the outer envelope and surrounding soft tissues is clear, which provides favorable conditions for ultrasound diagnosis. The self-regulation of thyroid function refers to the regulation of the secretion of thyroxine by the amount of iodine supplied by the thyroid itself in the absence of TSH or the concentration of TSH is unchanged. Therefore, for the identification and diagnosis of benign and malignant thyroid nodules, ultrasound has always been one of the preferred imaging methods. With the continuous improvement of the level of science and technology, ultrasound inspection technology has also improved. When using ultrasound to diagnose thyroid diseases, thyroid neoplastic lesions can be displayed more clearly on the ultrasound images, and the lesions can be found in time and medical measures can be taken to control the condition. However, thyroid diseases are complex and changeable, especially malignant thyroid nodules, which are difficult to diagnose and control. During an ultrasound examination, benign and malignant nodules overlap on the two-dimensional sound image, which makes the diagnosis more difficult. Especially when some nodules have both benign and malignant characteristics, it is difficult to distinguish and qualitatively diagnose their nature based on the sonogram alone, which directly affects the choice of clinical treatment and surgical methods. This puts forward higher requirements for the initial qualitative diagnosis of lesion formation for ultrasound diagnosticians. Therefore, medicine urgently needs more advanced ultrasound diagnostic technology to overcome the difficulties encountered when using conventional ultrasound examination methods to diagnose thyroid diseases so as to help clinicians better diagnose and treat thyroid diseases and protect the health of patients. There is a clinical need for an intelligent diagnosis technology of thyroid diseases based on ultrasound images, which can provide objective and reliable auxiliary diagnosis opinions for thyroid diseases through the texture, shape, and other information of the images, freeing doctors from heavy work.

Because few patients with diffuse thyroid disease participated in a tissue biopsy, and it was difficult to obtain patient data, there are few researches on the intelligent diagnosis of diffuse thyroid disease at home and abroad. There have been many studies on diagnostic methods of thyroid diseases in academic circles today. Among them, Omiotek's research conducted thyroid ultrasound image analysis and analyzed the close relationship between thyroid nodule lesions and ultrasound image texture under the diffuse form of Hashimoto's thyroid disease. His research obtained a set of nine fractal descriptors of thyroid ultrasound images, which can distinguish healthy cases from patients with diffuse Hashimoto's thyroiditis [1]; Omiotek's research aims to build an effective classifier that automatically recognizes and classifies ultrasound images of the thyroid gland to detect cases affected by Hashimoto's thyroid gland. In the research, he used 10 supervised learning techniques and the majority vote of the combined classifier, and the result of the classifier obtained proposed two thyroid ultrasound detection models with a sensitivity of 88.1% [2]. Chen's research focuses on the study of thyroid bimodal and multimodal imaging systems. In the research, he obtained a kind of dual-modal fluorescence/computed tomography (CT) gold iodide nanoclusters that can be used to visualize malignant thyroid cancer through relevant experimental analysis. This multimodal cluster can help achieve more accurate image capture of malignant thyroid nodules, thereby improving the timeliness and effectiveness of the diagnosis of malignant thyroid nodules [3]; Sorrenti S's research puts forward that the current difficulty in diagnosing thyroid diseases is the improvement in the ability of inaccessible small thyroid nodules to become malignant. Therefore, the main focus of his research is to develop new molecular methods to improve the diagnosis of malignant thyroid nodules, and he has made great progress in the potential molecular mechanisms of deregulation [4]. Qin's research is based on the starting point of effectively using the features of thyroid ultrasound images and proposes a combination of traditional ultrasound and ultrasound elastography based on convolutional neural networks. This introduces richer characteristic information for the classification of benign and malignant thyroid nodules to help diagnose benign and malignant thyroid nodules [5]. Lai's research carried out the current commonly used thyroid imaging report and data system, namely the accuracy comparison of ACR TI-RADS and Kwak TI-RADS in the diagnosis of thyroid benign and malignant nodules, and concluded that ACR TI-RADS and Kwak TI-RADS have good accuracy in the differential diagnosis of thyroid nodules, but ACR TI-RADS has a higher specificity and a lower sensitivity than Kwak TI-RADS [6].

The above studies are all based on the analysis and research of thyroid disease diagnosis, and methods or conclusions have been drawn that can be used to overcome thyroid disease diagnosis. However, the experimental process of these studies is more complicated and requires a lot of time and energy. The innovation of this article lies in the simple and reliable pathological study of thyroid cases combined with SMI technology and contrast-enhanced ultrasound. This article uses machine learning methods to achieve quantitative description of different diseases through the design features of ultrasonic images of diffuse diseases and finally realizes the diagnosis of diffuse diseases. It concludes that SMI technology and contrast-enhanced ultrasound examination have good diagnostic efficiency and high application value in the identification and diagnosis of benign and malignant thyroid nodules.

## 2. Diagnosis of Benign and Malignant Thyroid Nodules

### 2.1. SMI Technology

#### 2.1.1. SMI Technology Principle

SMI technology (superb microvascular imaging technology) is a new ultrasound diagnostic imaging method proposed by Canon in Japan in 2014. The principle basis of SMI technology is the motion suppression technology used to isolate and eliminate clutter but retain the vulgar blood flow signal. It includes ultrasound diagnostics, ultrasound therapy, and biomedical ultrasound engineering. Therefore, ultrasound medicine has the characteristics of combining medicine, science, and engineering. It involves a wide range of contents and has a high value in the prevention, diagnosis, and treatment of diseases. In the motion suppression technology, the ultrasonic detection image subtracts the change of the structure position from one frame to another, leaving only the color imaging part. SMI technology uses an adaptive wall wave to suppress clutter noise and minimize the flash artifacts of the image. There are two imaging methods for SMI technology: monochrome mode and color mode [7]. Monochrome mode only focuses on the vascular system and improves the sensitivity to the vascular system by suppressing its background signal, and the output result is a grayscale image; the color mode provides both grayscale and color images. The examination of thyroid nodules generally includes thyroid B-ultrasound, thyroid radionuclide scan, neck X-ray examination, thyroid fine-needle aspiration cytology examination, thyroid function test, etc. SMI technology can detect very low blood flow in the lesion and can noninvasively and truly reflect the blood perfusion state of the nodule. With the widespread application of ultrasound technology, SMI technology has now become one of the important methods for the identification and diagnosis of benign and malignant thyroid nodules [8]. The SMI technology display is shown in Figure 1.

#### 2.1.2. SMI Algorithm (Sampling Matrix Inversion Algorithm)

Another name for the SMI algorithm is the matrix inversion algorithm. It calculates the weight vector directly according to the estimated sampling covariance matrix inversion, which can overcome the influence of the eigenvalue score of the covariance matrix on the weight vector. Thus improving the data processing speed [9]. The algorithm satisfies the maximum signal-to-noise ratio criterion:

(1) $$\begin{array}{c} \text{Max SINR}=\max\left(W^{h}R_{s}W\right)W^{h}R_{n+1}, \end{array}$$

where *R*_*n*+1_ is the inverse of the interference noise covariance matrix, *R*_*s*_ is the desired signal covariance matrix, and *W* is the adaptive weight vector. The optimal weight vector can be expressed as follows:

(2) $$\begin{array}{c} W_{p}=aR_{n+1}\theta_{o}, \end{array}$$

where *R*_*n*+1_ is the noise ratio of the interference covariance matrix, and *θ*_*o*_ is the steering vector of the signal. In fact, the signal, beam, and interference environment and their statistical characteristics are often known a priori. The exact value of *R*_*n*+1_ cannot be obtained, but it is assumed that the signal, clutter, and interference are all statistically stable or partially stable. According to the time stability of the signal, the maximum likelihood estimate can be obtained from the snapshot data:

(3) $$\begin{array}{c} R_{I}=K^{-1}\sum_{k=1}^{K}X_{i}kX_{n}K, \end{array}$$

where *R*_*i*_ is the interference noise covariance matrix, and the adaptive vector of the SMI algorithm is as follows:

(4) $$\begin{array}{c} W_{i}=R_{i+n}a\vartheta_{O}\left(R_{i+n}a\right), \end{array}$$

where *W*_*i*_ is the desired adaptive vector, which is directly related to the similarity of the actual value and the magnitude of the estimated variance. Therefore, a deviation between the estimation of the covariance matrix and the actual value will inevitably occur, which will cause the diffusion of the eigenvalues, which will lead to adaptive beam distortion, and which seriously affects the performance of the beam [10]. Taking the eigenvalue *F*, the estimation of the interference noise covariance matrix is as follows:

(5) $$\begin{array}{c} R_{i+n}=\frac{1}{f}\sum_{f=1}^{n}X_{i+n}\left(nK+k\right)X_{i+n}. \end{array}$$

According to the size of the interference noise frequency and the radar sampling frequency, *n* is the appropriate step length, and *K* is the signal window length. The data are sampled in a window with a step length of *n*, and the interference noise covariance matrix is estimated multiple times from the taken data:

(6) $$\begin{array}{c} R_{i+n}=K^{-1}\sum_{k=1}^{x}X_{i+n}\left(N+K\right)X_{n-i}, \end{array}$$

where *X* is the step length whose value is appropriately increased. To obtain the estimated interference covariance matrix, the average value is taken, and the obtained covariance matrix has a certain statistical significance. When the sampled data are small, the adaptive beam sidelobe is very high, which reduces the performance of the maximum output signal dryness ratio. At this time, the SINR corresponding to the optimal weight vector of the matrix is as follows:

(7) $$\begin{array}{c} \text{SINR}=WR_{s}W\left(WR_{i+n}\right). \end{array}$$

When the performance of the adaptive beamformer is lower than that of the optimal beamformer, the SINR loss caused is recorded as follows:

(8) $$\begin{array}{c} L=\text{SINR}\left(W{\text{SINR}}_{i}\right)K, \end{array}$$

where *SINR*_*i*_ is the optimal weight vector of the matrix corresponding to the output signal dryness ratio; *L* is the SINR loss; and the smaller the *SINR*_*i*_, the larger the *L*, which means the more serious the loss, the worse the performance, and vice versa. The basic flow of the SMI algorithm is shown in Figure 2.

### 2.2. Contrast-Enhanced Ultrasound Examination

#### 2.2.1. The Principle of Contrast-Enhanced Ultrasound Detection

Ultrasound technology is a high-tech developed in the 20th century. It is an emerging, interdisciplinary, and borderline science, which has attracted extensive attention of scientific and technological workers in countries such as the United States, Germany, Canada, Japan, and China. Contrast-enhanced ultrasound technology is a very prominent technological development in the field of ultrasound imaging diagnostics in recent years, and it can also be called the third leapfrogging revolution in the history of ultrasound imaging. Contrast-enhanced ultrasound uses low mechanical index (MI0.2) pulse contrast sequence imaging technology for ultrasound inspection, so it reduces the damage to microbubbles and greatly improves the signal-to-noise ratio of the image. It can show the fine blood circulation process of the nodule tissue and its vascular perfusion, thereby improving the detection rate of the lesion and completing the dynamic observation of the whole process of the perfusion of the contrast agent in the lesion [11]. With the development of contrast-enhanced ultrasound examination technology, contrast-enhanced ultrasound has begun to enter the stage of clinical treatment application. Contrast-enhanced ultrasound can also significantly improve the ability to monitor blood flow information around the mass, thereby helping to identify and treat benign and malignant nodules around the thyroid. At the same time, contrast-enhanced ultrasound technology can also complete the entire observation of blood flow distribution and blood perfusion around thyroid nodules. Also, the possibility of displaying the tumor microvascular perfusion process and the full-view imaging display of tumor neovascularization is improved so as to provide a new method for evaluating the benign and malignant quality of thyroid nodules [12].

#### 2.2.2. Contrast-Enhanced Ultrasound Exercise Correction Method

In the project of acquiring a dynamic image by contrast-enhanced ultrasound, although the detected object can hold the breath for a short time, the slight movement of the organs cannot be completely eliminated, and the organ movement may be more serious after the breath-hold is over. In order to comprehensively use multiple imaging modes or co-modal changes to provide more complete information, the ultrasound contrast motion correction algorithm often integrates all effective information to make up for information deficiencies and better serve clinical diagnosis and treatment. The most important step of integration is to make the geometric positions reached by multiple images in the spatial domain completely correspond; this step is called registration [13]. Registration refers to the matching of geographic coordinates of different image patterns obtained by different imaging methods in the same area, including geometric correction, projection transformation, and unified scale processing.

Mutual information registration is the main step of registration. It refers to the statistical correlation of information between two radiographic pictures. The formula for mutual information registration is as follows:

(9) $$\begin{array}{c} F\left(A,B\right)=H\left(A\right)+H\left(B\right)-H\left(A,B\right), \end{array}$$

where

(10) $$\begin{array}{c} F\left(A,B\right)=H\left(A\right)-H\left(\frac{A}{B}\right). \end{array}$$

At last,

(11) $$\begin{array}{c} F\left(A,B\right)=H\left(B\right)-H\left(\frac{B}{A}\right), \end{array}$$

where *A* and *B* refer to two different contrast pictures. For an image, *H* represents the amount of information of this image. The definition formula is as follows:

(12) $$\begin{array}{c} H\left(A\right)=\sum_{a}P_{A}\left(a\right)\text{log}P_{A}. \end{array}$$

And the joint set of the two images is

(13) $$\begin{array}{c} H\left(A,B\right)=\sum_{P_{A}}\left(a,b\right)\text{log}P_{AB}\left(a,b\right). \end{array}$$

Mutual information registration is based on the following principle: when two images based on a common anatomical structure reach the optimal registration value, the mutual information of their corresponding image features should be the maximum, which is

(14) $$\begin{array}{c} a=\arg.\max I\left(A,B\right), \end{array}$$

where *a* is the misregistration function, (*A*, *B*) is a set of mutual information, and mutual information *l*(*A*, *B*) as the similarity measure of the registration of two images must satisfy a condition: If it cannot fluctuate with the change of the mismatch function *a*, it will lead to the generation of local extrema during the registration process.

From the current point of view, there are two ways of grayscale testing. One is the grayscale test release system built into the software system, and the other is to use third-party tools to assist in the implementation. Both methods are feasible. In order to avoid the extreme value of mutual information and increase the speed of calculation, the main shaft moment registration algorithm in the registration method can be used for registration. The principal axis moment registration algorithm converts the gray content of an image into a geometric representation of quantity and direction [14, 15]. Regarding the gray value of each pixel in the two images as the quality of the pixel, the centroid of the image is calculated by the classical mechanics calculation method as shown in the following formula:

(15) $$\begin{array}{c} X_{c}=\sum_{i=1}^{n}x_{i}P_{i},\\ Y_{c}=\sum_{i=1}^{n}y_{i}p_{i}, \end{array}$$

where *X*_*i*_ and *y*_*i*_ represent the coordinates of the pixel, *P*_*i*_ represents the gray value of the pixel, and *n* represents the number of pixels in the image. The spindle moment algorithm can solve the problem of easily falling into the local optimal value and effectively improve the accuracy and speed of ultrasound contrast registration [16] (Figure 3).

## 3. Diagnosis Test of Thyroid Benign and Malignant Nodules

### 3.1. Experimental Method

The experimental methods of this study are as follows: first, 40 cases of benign and malignant thyroid nodules in China in 2018 were randomly selected. Among them, there were 20 cases of benign and malignant nodules. The maximum diameter of the nodules was 0.6∼3.9 cm, with an average of 2.10.3 cm. The pathological results of all nodules were obtained through fine-needle aspiration biopsy or surgical treatment. Then, according to the standard blood flow distribution pattern of thyroid nodules, SMI technology and contrast-enhanced ultrasound were used to judge, and two different selected nodule cases composed of 20 nodules in each group (10 benign and malignant nodules) compared the distribution pattern of blood flow and the morphological characteristics of blood vessels. Finally, through ROC curve calculation and analysis, the specificity and sensitivity of the two diagnostic methods for pathological diagnosis are obtained so as to evaluate and compare the diagnostic efficiency and application value of the two diagnostic methods of SMI and contrast-enhanced ultrasound. Lower specificity and higher sensitivity of the diagnosis method will have a better diagnostic effect and application value of thyroid benign and malignant nodules. The standard blood flow distribution pattern of thyroid nodules is: if there is no blood signal on the periphery and inside of the nodule, it is judged as no blood flow type; if the nodule shows the main part of peripheral blood flow, it is judged as peripheral blood flow; if the nodule shows the main part of internal blood, it is judged as central blood flow; and if there are abundant blood flow signals inside and around the nodule, it is judged as mixed blood flow [17].

### 3.2. SMI Technical Diagnosis

#### 3.2.1. SMI Ultrasound Examination Results

Before evaluating the blood flow pattern and vascular morphological characteristics of SMI nodules, an ultrasound examination of SMI nodules is performed first to grasp the pathology. The inspection results are shown in Table 1.

It can be seen from the results of the above table that SMI nodule ultrasound examination is accurate for different types of benign and malignant nodules. It is feasible to use SMI technology to diagnose thyroid nodules.

#### 3.2.2. Nodule Blood Flow Distribution Pattern and Vascular Morphological Characteristics under SMI Technology

According to the standard blood flow distribution pattern of thyroid nodules, in this experiment, SMI technology was used to judge the blood flow distribution pattern of nodules 4 times. After 4 judgments, the results of the nodule blood flow distribution pattern are shown in Figure 4.

It can be seen from the results in Figure 4 that the analysis of the blood flow distribution pattern of SMI technical nodules in 20 cases of benign and malignant thyroid nodules in this group showed that the number of central and mixed nodules was the same, and the number of peripheral nodules was the least. After evaluation, through 4 repeated judgments, the blood flow distribution pattern of the nodules under SMI technology is completely consistent with the actual case. It shows that SMI technology has a high accuracy rate for displaying the blood flow distribution pattern of thyroid nodules. Next, let us look at the vascular morphological characteristics of the case nodules under SMI technology. Because the vascular morphological characteristics of benign nodules are mainly linear and branched under ultrasound detection, the shape of the same thickness is not comparable. Therefore, the SMI microvascular imaging cases extracted in this experiment are all cases of malignant thyroid nodules. SMI angiography showed that the vascular morphology of malignant nodules was stump type and crab foot type, with more tortuous and chaotic directions, and more irregular small branches, which was in line with the actual situation. This shows that SMI technology has a good imaging effect on nodular blood vessels.

In summary, SMI technology has good diagnostic efficiency for benign and malignant thyroid nodules.

### 3.3. Contrast-Enhanced Ultrasound Diagnosis

#### 3.3.1. Ultrasonic Examination Results

Similarly, before evaluating the blood flow distribution pattern and vascular morphological characteristics of the nodules under ultrasound detection, we also need to first perform contrast-enhanced ultrasound case inspection to grasp the pathology from the perspective of contrast-enhanced ultrasound detection. Ultrasonic contrast (ultrasonic contrast), also known as acoustic contrast, is a technique that uses a contrast agent to enhance the backscattered echoes and significantly improve the resolution, sensitivity, and specificity of ultrasound diagnosis. The results of contrast-enhanced ultrasound examination of benign and malignant nodules in 20 thyroid cases in this experiment are shown in Table 2.

From Table 2, we can see that the contrast-enhanced ultrasound examination is accurate in the diagnosis of various types of benign and malignant nodules in the case. However, compared with SMI technology ultrasound diagnosis, the diagnostic accuracy of contrast-enhanced ultrasound examination is slightly lower. It shows that the use of contrast-enhanced ultrasound to diagnose benign and malignant thyroid nodules is also feasible, but the effect is slightly inferior to SMI technology. Chinese medicine believes that it is mainly due to the close relationship between emotional internal injury, diet, unsuitable soil and water, and congenital factors.

#### 3.3.2. Blood Flow Distribution Pattern and Vascular Morphological Characteristics of Nodules under Contrast-Enhanced Ultrasound

Thyroid nodules can be single or multiple. The incidence of multiple nodules is higher than that of single nodules. According to the standard blood flow distribution pattern of thyroid nodules, in this experiment, the same contrast-enhanced ultrasound was used to judge the blood flow distribution pattern of the nodules 4 times. After 4 judgments, the results of the nodule blood flow distribution pattern are shown in Figure 5.

From the results shown in Figure 5, we can see that contrast-enhanced ultrasound examination of 20 cases of benign and malignant thyroid nodules in this group showed the blood flow distribution pattern of the nodules. The number of peripheral and mixed nodules is not much different, and the results of the 4 inspections are relatively stable. The number of central nodules is the largest, and the results of the 4 inspections are slightly fluctuating. This result after evaluation shows that: contrast-enhanced ultrasound examination has certain accuracy in judging the blood flow distribution pattern of thyroid nodules, but there are still some errors. This also shows that the accuracy of contrast-enhanced ultrasound in judging the blood flow distribution pattern of thyroid nodules is slightly lower than that of SMI technology [18].

Next, let us look at the vascular morphological characteristics of 20 benign and malignant thyroid nodules in this group under the state of contrast-enhanced ultrasound. In the same way, the vascular imaging cases taken this time by ultrasound imaging are also malignant nodules. Because in the ultrasound imaging of blood vessels, the vascular morphology of benign nodules is mainly linear and branched, and the shape of the same thickness is still not comparable [19]. Under contrast-enhanced ultrasound detection, we observed that the vascular morphology of malignant nodules has many small branches and microvascular details, and the vascular movement is disorderly, mainly in the form of cynopods. This is consistent with the actual situation of the nodular blood vessel morphology of the selected malignant nodule cases, indicating that the contrast-enhanced ultrasound examination also has a better imaging effect on nodular blood vessels.

In summary, it can be concluded that contrast-enhanced ultrasound has a certain diagnostic power for benign and malignant thyroid nodules, but its diagnostic power is slightly insufficient compared with the diagnostic power of SMI technology.

### 3.4. Comparison of Specificity and Sensitivity

After the conclusion of the blood flow distribution pattern and blood vessel morphology of SMI technology and contrast-enhanced ultrasound examination, the last step of this experiment will be carried out next, that is combining the blood flow distribution pattern and the result of the blood vessel morphology judgment. They used ROC curves to calculate the specificity and sensitivity of SMI technology and contrast-enhanced ultrasound in the identification and diagnosis of benign and malignant thyroid nodules. The RI value calculated using the ROC curve represents the best diagnostic point for distinguishing benign and malignant thyroid nodules in SMI and contrast-enhanced ultrasound modes, that is the best diagnostic sensitivity. According to the pathological diagnostic criteria, the area of the upper part of the corresponding curve is the diagnostic specificity [20]. The ROC curve calculation results of SMI technology and contrast-enhanced ultrasound examination are shown in Figure 6.

From Figure 6, the ROC curve calculation results of SMI and contrast-enhanced ultrasound are as follows: the final RI value of SMI is the diagnostic sensitivity, which is 0.83 and the specificity is 0.24; the final RI value of contrast-enhanced ultrasound is 0.81, that is the diagnostic sensitivity is 0.81 and the specificity is 0.26. It can be seen that although the ROC curve calculation results of SMI technology and contrast-enhanced ultrasound examination are not much different, there are still slight differences. That is, when the sensitivity of the two diagnostic techniques is high, the diagnostic sensitivity of SMI technology is slightly higher than that of contrast-enhanced ultrasound, and the diagnostic specificity of contrast-enhanced ultrasound is slightly higher than that of SMI. This result shows that SMI technology and contrast-enhanced ultrasound examination have certain diagnostic efficiency and application value for the diagnosis of benign and malignant thyroid nodules, but the diagnostic efficiency and application value of SMI technology is slightly higher than that of contrast-enhanced ultrasound examination [21–24].

## 4. Discussion

The correct identification and diagnosis of thyroid benign and malignant nodules are of great significance to the treatment of thyroid diseases. Conventional ultrasound examination is currently the most commonly used examination method for thyroid diseases. It is noninvasive and highly useable and can quickly and clearly differentiate and diagnose benign and malignant thyroid nodules. But at the same time, it also has certain limitations, such as images sometimes overlap. This will directly affect the diagnosis and treatment of thyroid diseases. Therefore, this article designs a diagnostic experiment for benign and malignant thyroid nodules based on SMI technology and contrast-enhanced ultrasound, aiming to explore the application value of SMI technology and contrast-enhanced ultrasound in the diagnosis of thyroid diseases. In the above experiment, the selected 40 cases of thyroid benign and malignant nodules were diagnosed by SMI technology and contrast-enhanced ultrasound examination to determine the blood flow distribution patterns and vascular morphological characteristics in the two diagnostic modes. And evaluating its correct rate and using the ROC curve to calculate the diagnostic sensitivity and specificity of these two diagnostic techniques [25], the following conclusions are drawn: for the judgment of blood flow distribution pattern and vascular morphological characteristics, the judgment accuracy rate of SMI technology is slightly higher than that of contrast-enhanced ultrasound examination; as for the diagnostic specificity and sensitivity, the sensitivity of the two diagnostic techniques is higher. The diagnostic sensitivity of contrast-enhanced ultrasound is slightly lower than that of SMI technology, and the specificity is slightly higher than that of SMI technology. This conclusion shows that both the SMI technique and the contrast-enhanced ultrasound examination have good diagnostic efficiency and application value for benign and malignant thyroid nodules. In general, the diagnostic efficiency and application value of SMI technology is better than that of contrast-enhanced ultrasound. The results of this experiment show that SMI technology and contrast-enhanced ultrasound have improved the diagnostic performance of benign and malignant thyroid nodules based on traditional ultrasound detection technology. They have higher diagnostic sensitivity, that is better diagnostic results. It shows that the application of SMI technology and contrast-enhanced ultrasound in the diagnosis of thyroid benign and malignant nodules has a certain application value. With the continuous development and progress of science and technology, SMI technology and contrast-enhanced ultrasound examination will inevitably continue to update and progress so as to better serve the diagnosis of thyroid benign and malignant nodules and promote the diagnosis and clinical treatment of thyroid diseases.

## 5. Conclusions

With the improvement of medical technology in today's society and the enhancement of people's health awareness, people's attention to thyroid diseases continues to increase. However, thyroid diseases, such as malignant secretory tumor diseases, are more complex and changeable, especially for malignant thyroid nodules, which are difficult in clinical diagnosis and treatment. Conventional thyroid ultrasound examination methods also have certain limitations, such as: for benign and malignant thyroid lesions, two-dimensional detection images sometimes overlap, which can also lead to different images of the same disease, and the same frequency of different diseases; at the same time, the blood flow with a low flow rate will not be displayed. And usually, it can only clearly display the larger blood vessel images, but the new microvascular network of the tumor cannot show its full picture, which means that thyroid cancer with less blood supply is easy to be missed. These deficiencies in conventional ultrasound examinations will directly affect the clinical treatment of thyroid diseases. Therefore, the medical field of thyroid diseases urgently needs more advanced ultrasound diagnostic technology to overcome the difficulties encountered in the diagnosis of thyroid diseases so as to help clinicians better diagnose and treat thyroid diseases and protect the health of patients. With the improvement of science and technology, two more advanced ultrasound detection technologies, SMI technology and contrast-enhanced ultrasound, have emerged in medicine. SMI technology can detect very low blood flow in thyroid lesions and can noninvasively and truly reflect the blood perfusion state of the nodules; contrast-enhanced ultrasound can continuously and dynamically observe the vascular distribution and blood perfusion of thyroid nodules, showing that the possibility of tumor neovascularization has also been improved. Therefore, SMI technology and contrast-enhanced ultrasound technology can solve the current problems in the diagnosis and treatment of thyroid diseases to a certain extent by virtue of their own advantages and have begun to be used in the identification and diagnosis of thyroid benign and malignant nodules. The research in this article has proved through experiments that SMI technology and contrast-enhanced ultrasound have high diagnostic sensitivity for the identification and diagnosis of benign and malignant thyroid nodules, that is they have better diagnostic efficiency and application value. And from the comparison of sensitivity, the diagnostic sensitivity of SMI technology is slightly higher than that of contrast-enhanced ultrasound, which shows that SMI technology has slightly better diagnostic performance and application value than contrast-enhanced ultrasound. The findings of this article provide a meaningful reference for the medical community to better apply SMI technology and contrast-enhanced ultrasound in the diagnosis and treatment of thyroid diseases. The number of features extracted manually in the research of thyroid nodular disease in this article is relatively small. In the future, more features can be added to study the interaction between artificial features and neural network features to achieve better classification results.

## Figures and Tables

**Figure 1:** SMI technology display.

**Figure 2:** The basic flow of the SMI algorithm.

**Figure 3:** The basic flow of the contrast-enhanced ultrasound motion correction algorithm.

**Figure 4:** Nodule blood flow distribution pattern in SMI technology. (a) Statistics of the number of SMI blood flow distribution patterns. (b) Proportion of SMI blood flow distribution patterns.

**Figure 5:** Contrast-enhanced ultrasound examination of nodule blood flow distribution pattern. (a) Statistics of the number of blood flow distribution patterns (b). Proportion of blood flow distribution patterns.

**Figure 6:** ROC curve of SMI and contrast-enhanced ultrasound.

**Table 1:** Ultrasonography results of SMI nodules.

ACR TI-RADS classification	Benign	Malignant	Predicted malignancy rate	Actual malignancy rate (%)
TR3	4	3	<20%	15
TR4	4	3	<20%	15
TR5	2	4	>30%	40

Note. ACR TI-RADS, American Society of Radiology Thyroid Imaging Report and Data System.

**Table 2:** Results of contrast-enhanced ultrasound nodules.

ACR ti-RADS classification	Benign	Malignant	Predicted malignancy rate	Actual malignancy rate (%)
TR3	5	2	<20%	10
TR4	3	4	<30%	20
TR5	2	4	>10%	20

## Data Availability

The data that support the findings of this study are available from the corresponding author upon reasonable request.
